The article "Privacy Protection of Healthcare Data over Social Networks Using Machine Learning Algorithms" was retracted in 2023. Reasons: signs of a paper mill; suspected computer-generated content; unreliable results or conclusions; concerns about the data.

# Privacy Protection of Healthcare Data over Social Networks Using Machine Learning Algorithms

**DOI:** 10.1155/2022/9985933

**Published:** 2022-03-24

**Authors:** Shakir Khan, V. Saravanan, Gnanaprakasam C. N, T. Jaya Lakshmi, Nabamita Deb, Nashwan Adnan Othman

**Affiliations:** ^1^College of Computer and Information Sciences, Imam Mohammad Ibn Saud Islamic University (IMSIU), Riyadh, Saudi Arabia; ^2^Department of Computer Science, College of Engineering and Technology, Dambi Dollo University, Dambi Dollo, Oromia Region, Ethiopia; ^3^Department of Electronics and Instrumentation Engineering, St. Joseph's College of Engineering, Chennai 600119, Tamilnadu, India; ^4^Department of Computer Science and Engineering, SRM University, Amaravati, AP, India; ^5^Department of Information Technology, Gauhati University, Gawahati, Assam 781014, India; ^6^Department of Computer Science, College of Science, Knowledge University, Erbil 44001, Iraq

## Abstract

With the rapid development of mobile medical care, medical institutions also have the hidden danger of privacy leakage while sharing personal medical data. Based on the k-anonymity and l-diversity supervised models, it is proposed to use the classified personalized entropy l-diversity privacy protection model to protect user privacy in a fine-grained manner. By distinguishing solid and weak sensitive attribute values, the constraints on sensitive attributes are improved, and the sensitive information is reduced for the leakage probability of vital information to achieve the safety of medical data sharing. This research offers a customized information entropy l-diversity model and performs experiments to tackle the issues that the information entropy l-diversity model does not discriminate between strong and weak sensitive features. Data analysis and experimental results show that this method can minimize execution time while improving data accuracy and service quality, which is more effective than existing solutions. The limits of solid and weak on sensitive qualities are enhanced, sensitive data are reduced, and the chance of crucial data leakage is lowered, all of which contribute to the security of healthcare data exchange. This research offers a customized information entropy l-diversity model and performs experiments to tackle the issues that the information entropy l-diversity model does not discriminate between strong and weak sensitive features. The scope of this research is that this paper enhances data accuracy while minimizing the algorithm's execution time.

## 1. Introduction

With the rapid development of mobile medical technology, the gradual expansion of medical data sharing, and the continuous updating of data mining technology and deep learning technology, the sharing of medical data between different hospitals has become more convenient. The mining and sharing data and information also create enormous economic and social values. However, a problem cannot be ignored in data release and sharing. To calculate the anonymous cost, this article presents a technique based on the extension level. The different aggregate levels of the attribute must be built first. That is, the privacy of medical patients is leaked. If medical institutions do not fully consider data privacy issues when sharing data, illegal users (attackers) can use data released by other institutions to speculate in series or even use data vulnerabilities released by the same hospital at different times to obtain medical patients' privacy sensitivity and information, thereby causing an unpredictable risk of leakage to patient privacy. In the past, when medical institutions shared or released medical data for privacy protection, they would choose to remove some personal identification information, such as name, address, and phone number. However, attackers can still obtain some insensitive user information through other means. For example, this information is used to correspond with the user's disease diagnosis data to get the patient's privacy about the disease. This attack is also called a link attack [1].

Table 1 is a medical datasheet. The hospital did not explicitly give the patient's name when released. However, assuming that the attacker obtains the voting table of the voters in the user's jurisdiction, as shown in Table 2 on the network, the attacker can link the common attributes of the two tables, such as zip code (430056), to infer the patient's status, name (Kevin), and the disease “overweight.” If an evil attacker sells this information to a weight loss center, it will directly leak the patient's (Kevin) private information.

This research paper is organized as follows: Section 1 describes the introduction. The privacy protection based on the principle of anonymity is described in Section 2.  Section 3 describes the information entropy I-diversity model. The personalized information entropy is described in Section 4.  Section 5 describes experimental results and analysis. The conclusion is described in Section 6.

## 2. Privacy Protection Based on the Principle of Anonymity

Privacy protection based on the principle of anonymity mainly processes the relevant attributes in the data table through technical means, such as data generalization and data suppression [2, 3], before data are released or shared and do not release or restrict the release of specific data. In this way, personal identification information loses association with sensitive attributes and achieves the purpose of privacy protection [4, 5]. Researchers are also proposing various security protocols for keeping the information confidential and secure which is shared among the users and servers in wireless network using several IoT devices [6].

### 2.1. k-Anonymous Thought

Among the many privacy protection methods based on the anonymity principle, k-anonymity has become a necessary technical means for privacy protection in data release because it protects private information while ensuring data availability [7, 8]. The core idea is to publish low-precision data through generalization and concealment techniques. Each record has at least the same quasi identifier attribute value as the other *k* − 1 data in the data table, reducing privacy caused by link attacks leakage [9].

**Definition 1 .**

k-anonymity: given a data table *U* {*B*_1_, *B*_2_,…, *B*_*n*_}, the quasi-identifier of *U* is RI, if and only if each value sequence in *U*[RI] in *U*[RI] appears at least *k* times. It is said that table *U* satisfies k-anonymity on QI. *T* [QI] represents the projection of the tuple of table *U* on RI.

### 2.2. k-Anonymity

The essence of k-anonymity requires that every record in the dataset has the same projection on the quasi identifier with at least *k* − 1 records. Therefore, the probability that the form where an individual is located is determined that does not exceed 1 *k*. Generalization [10] is a technical way to achieve anonymized privacy protection. Its essence is to replace specific values with generalized values or intervals and increase attackers' difficulty in obtaining individual private information by reducing data accuracy.  Table 3 is an anonymous medical data table satisfying *k* = 2 after generalization.

### 2.3. k-Anonymity Disadvantages

Although the k-anonymity algorithm improves the security of published information, it loses part of the data availability due to the need to generalize and conceal specific attributes of the data table. At the same time, the k-anonymity algorithm has the disadvantage of inaccurate query results during the calculation process, especially in the scenario where users are scarce. In addition, it will generate a larger anonymous area, thereby increasing the communication overhead.

## 3. Information Entropy l-Diversity Model

The generalized data table satisfies k-anonymity, which ensures that a particular user is in the set of *k* individuals of the same category so that individual users with the same quasi identifier are indistinguishable, thereby achieving a certain degree of anonymity protection. However, we suppose that *k* tuples in the same equivalence class have the same value on the sensitive attributes. Because it preserves private information while preserving availability of data, k-anonymity has now become a necessary technical technique for privacy protection in data release. The main concept is to use generalization and concealing methods to release low-precision data. Every record in the datasheet seems to have at least the very same quasi-identifier parameter value as the other *k* − 1 data, limiting privacy risks caused by link threats. The advantages of this algorithm are that the k-anonymity technique increases the privacy of released information; it reduces the data accessibility by requiring the generalizations and concealment of certain data table properties. In that case, the individual user records will be attacked by homogeneity and cause attribute leakage, such as the second equivalence class in Table 3.

To solve the privacy leakage problem caused by homogeneity attacks, literature [11] proposes the *l*-diversity model, which requires each equivalence class to contain at least *l* well-presented sensitivities. Attribute value, taking into account the constraints on sensitive attributes. If each equivalence class in the data table has *l* different sensitive attribute values, then the data table is said to satisfy the *l*-diversity rule. Literature [7] also gives an information entropy l-diversity rule.

**Definition 2 .**

Entropy *l*-diversity: given a data table *U* {*B*_1_, *B*_2_,…, *B*_*n*_}, the quasi-identifier attribute is RI{*B*_*i*_, *B*_*i* + 1_,…, *B*_*j*_}, the sensitive attribute is TA, and *T* = {*T*_*i*_, *T*_*i* + 1_,…, *T*_j_} is the sensitive attribute value. Table *U* satisfies k-anonymity, and its equivalence class set is *F* = {*F*_1_, *F*_2_,…, *F*_*n*_}, if and only if for each equivalence class *F*_*i*_ = 1, 2,…, *n*⊆*F*, all satisfy. In formula (1), it is said that the data table *U* satisfies the information entropy *l*-diversity.

(1) $$\begin{array}{c} P\left(Ei,s\right)\mathrm{lg}P\left(Ei,s\right)\geq \mathrm{lg}\left(1\right), \end{array}$$

(2) $$\begin{array}{c} \sum_{t\in T}Q\left(F_{i},t\right)\mathrm{lg}Q\left(F_{i},t\right)\geq \mathrm{lg}\left(l\right). \end{array}$$

Among them, *Q*(*F*_*i*_, *t*) is the frequency of the sensitive attribute value *s* in the equivalence class *F*_*i*_; ∑_*t*∈*T*_*Q*(*F*_*i*_, *t*)lg*Q*(*F*_*i*_, *t*) is the information entropy of the equivalence class *F*_*i*_, also known as the information entropy diversity sex, denoted as entropy (*F*_*i*_). Information entropy reflects the distribution of attributes. The larger the information entropy, the more even the distribution of sensitive attribute values in the equivalence, and the more difficult it is to derive specific individuals. By type

(1) It can be seen that if the equivalence class satisfies the information entropy *l*-diversity, then the information entropy of the equivalence class is at least lg(*l*).  Table 4 is an equivalent class in the anonymous data table.

Table 4 shows that the information entropy *l*-diversity calculation results of an equivalence class are as follows:

(3) $$\begin{array}{c} \frac{4}{5}\mathrm{lg}\frac{4}{5}+\frac{1}{5}\mathrm{lg}+\frac{1}{5}\approx 0.217\approx \mathrm{lg}1.165. \end{array}$$

From the results, for the equivalence class, the diversity of information entropy is lg1.65, and the value of parameter *l* cannot exceed 1.65. Only one attribute can be taken, considering the definition of l-diversity. There is at least one different sensitive attribute value in the price category. For the published datasheet, this conclusion is obviously of little significance.

And 4 of the sensitive attributes in the equivalence class are “flu.” For many patients, this is not a sensitive attribute. We suppose that the equivalence class contains four sensitive details: “tuberculosis” sensitive points. Assuming that the attacker knows that someone is in the equivalence class, the attacker is confident to speculate that the person has the characteristics of “emphysema” disease tendency, which is unacceptable for the patient [12]. Medical information contains many nonsensitive attribute values such as “flu” or “fever,” and the disclosure of these attribute values will not infringe on individual privacy. Therefore, the information entropy l-diversity model does not distinguish between sensitive attribute values and cannot reflect the risk of privacy leakage in this case. This paper proposes a personalized information entropy *l*-diversity model to protect users' medical data privacy.

## 4. Personalized Information Entropy *l*-Diversity Model

### 4.1. Personalized Information Entropy

Diversity model definition has given the deficiencies of the information entropy *l*-diversity model; on the one hand, it is necessary to increase the information entropy value of the equivalence class. On the other hand, it is essential to distinguish sensitive attribute values and reduce information leakage with solid and sharp attributes.

Therefore, the sensitive attribute value can be divided into a robust and sensitive value SV (sensitive value) and a weak sensitive value DV (do not care value), modifying the information entropy l-diversity rule to obtain a new personalized information entropy l-diversity rule.

**Definition 3 .**

Personalized information entropy l-diversity: given a data table *U* {*B*_1_, *B*_2_,…, *B*_*n*_}, RI{*B*_*i*_, *B*_*i*+1_,…, *B*_*j*_} is the quasi identifier of *U*, and TA is the sensitive attribute, *T* = {*T*_*i*_, *T*_*i*+1_,…, *T*_*j*_} is the set of sensitive attribute values, SV represents the strong sensitivity value, DV is the weak sensitivity value, |SV| is the number of strong sensitivity values, |DV| is the weak sensitivity value Number. Table U satisfies k-anonymity, and its equivalence class set is *F* = {*F*_1_, *F*_2_,…, *F*_*n*_}, if and only if for each equivalence class *F*_*i*_ = 1, 2,…, *n*⊆*F*, all satisfy. In formula (2), it is said that the data table *U* satisfies the individualized information entropy *l*-diversity.

(4) $$\begin{array}{c} \frac{\left|DV\right|+\left|\text{SV}\right|}{\left|\text{SV}\right|}10^{\sum_{SV\in S}Q\left(F_{i},SV\right)\mathrm{lg}Q\left(F_{i},SV\right)}. \end{array}$$

Among them, *Q*(*F*_*i*_, SV) is the frequency of strong and sensitive attribute values appearing in the equivalence class. Rate |*DV*|+|SV|/|SV|10^∑_*SV*∈*S*_*Q*(*F*_*i*_, *SV*)*lgQ*(*F*_*i*_, *SV*)^ is the letter of personalized equivalence class diversity of information entropy.

It can be seen from formula (2) that it is necessary to calculate the frequency *Q*(*F*_*i*_, SV) of the susceptible attribute value in the equivalence class instead of calculating the weakly sensitive attribute value that will reduce the value of *Q*(*F*_*i*_, SV)lg*Q*(*F*_*i*_, SV) frequency of occurrence. Formula (2) is used to calculate the information entropy of the equivalence class in Table 4. There are DV = {flu}, SV = {emphysema}, |DV| = 1, |SV| = 1, and SV appears in the equivalence class. The probability is 1/5, and then the improved diversity of information entropy is

(5) $$\begin{array}{c} 1=1+1\;1\times 10-15\mathrm{lg}15\approx 2.2828,\\ m=\frac{1+1}{1}*10^{-\frac{1}{5}\mathrm{lg}\frac{1}{5}}\approx 2.2828. \end{array}$$

According to the calculation result, the value of *l* does not exceed 2.282 8. Then, *l* is 2, and the equivalence class satisfies 2-diversity. Personalized information entropy *l*-diversity is compared with information entropy *l*-diversity, it improves the information entropy of the equivalence class and reduces the correspondence between the private information and the identity information derived from the link in the equivalence class.

### 4.2. Information Loss Measurement

The anonymous privacy protection model based on k-anonymity and its improvement will inevitably produce information loss while protecting private information, which will affect data accuracy [13]. This is the anonymization cost. The anonymity cost is generated when the original data are generalized and suppressed in preprocessing operations. The anonymity cost measurement is an indicator to measure the information loss after the data is anonymized, and it can also judge the optimization degree of the anonymized dataset. The smaller the information loss, the greater the data accuracy, and higher is the data availability, and vice versa. Therefore, in the process of anonymization operation, the cost of anonymity should be reduced as much as possible.

This article adopts the method based on the generalization level to measure the anonymity cost and to use this method to measure the anonymity cost. It is necessary to construct the domain generalization level of the attribute. The amount of information in each layer in the domain generalization hierarchy is different. Generally, for the same quality, data at a higher level of generalization have less information than data at a lower level. It is calculated as follows:

(6) $$\begin{array}{c} \text{Qre}\left(ST\right)=1-\frac{\sum_{i=1}^{N}\sum_{j=1}^{N_{A}}h/\left|{\text{DGH}}_{Bi}\right|}{N*N_{A}}. \end{array}$$

Among them, *Qre* represents the accuracy of the data, which is the original data table; *ST* is the generalized data table; *N* means the number of attributes in the data table; *NA* is the number of records in the dataset; |DGH_*Bi*_| is the generalized hierarchical structure of the attribute *B*_*i*_ Height; *h* represents the height of the attribute *B*_*i*_ in the generalization hierarchy.

**Definition 4 .**

Domain generalization hierarchy: let *A* be the attribute of data table *U*; there is a function *f*_*h*_: *h* = 0, 1,…, *n* − 1 such that *B*_0_⟶^*h*_0_^*B*_1_⟶^*h*_1_^ ⋯ .⟶^*h*_*n*=1_^*B*_*n*_, and *B* = *B*_0_, |*B*_*n*_| = 1; then, the generalization domain layer of attribute **A** on *f*_*h*_: *h* = 0, 1,…, *n* − 1 can be expressed as ∪_*h*=0_^*n*^*h*, denoted as |DGH_*B*_ |.

{*A*_0_, *A*_1_, *A*_2_, *A*_3_} shows the bottom-up generalization process of Zip attributes, and each layer represents a generalization domain of the fact. As the DG keeps going up, the generalization degree of the quality gets higher and higher until it finally reaches the inhibited state. The generalization process is described as follows:

 
*A*_3_ = {^*∗∗∗∗∗*^}
  ↑
 
*A*_2_ = {021^*∗∗*^}
  ↑*Z*
 
*A*_1_ = {0213^*∗*^, 0214^*∗*^}
  ↑
 
*A*_0_ = {02138, 02139, 02141, 02142}

## 5. Experimental Results and Analysis

This experiment uses the incognito algorithm proposed in [14] to complete the anonymous operation process. The basic idea of the Incognito algorithm is to use global recoding technology to perform generalization operations on the original dataset in a bottom-up breadth-first manner, and at the same time, perform necessary pruning and iterative functions on the generalization graph to make the original dataset gradually optimize, to achieve anonymity effect. The main premise behind the incognito algorithm is to use worldwide recoding techniques to accomplish bottom-up breadth-first generalization operations on the entire dataset, while also performing required pruning and repetitive features on the generalization graph to progressively enhance the actual information set and achieve secrecy. With an adjustable sequence reduction limit, the incognito algorithm constructs a set of all potential k-anonymous full-domain extensions of *T*. The approach checks monosubsets of the quasi-identifier first, and iterates, testing k-anonymity with regard to considerably larger subsets, in a similar fashion of the subset characteristic. The program in this paper mainly considers the algorithm execution time and the information loss of the data table.

### 5.1. Experimental Data and Experimental Environment

The dataset used in the experiment is the Adult database in UCI [15], which is the most commonly used data source for k-anonymity research. The database has 32,206 pieces of data with a size of 5.5 MB, and the dataset contains a total of 15 attributes. We select eight attributes as the attribute set of quasi identifiers and select the Disease attribute as the sensitive attribute.  Table 5 describes the structure of the experimental dataset.

The experiment uses MySQL 5.5 to store data; the algorithm is implemented in Java; the experiment running environment is a 3.3 GHz Intel® Corei5 processor with 4 GB RAM.

We select Disease as the experimental sensitive attribute. The Disease attribute contains ten values, randomly generating disease types and using sensitivity weights to measure sensitivity [16]. The larger the value, the higher the sensitivity, as shown in Table 6. In the experiment, diseases with a sensitivity weight lower than 0.5 are set as weakly sensitive attributes.

### 5.2. Time Complexity Analysis

The solution in this paper first needs to calculate the personalized information entropy of the solid and sensitive value |SV| and the weak sensitive value |DV| diversity $\left|DV\right|+\left|\text{SV}\right|/\left|\text{SV}\right|10^{\sum_{SV\in S}Q\left(F_{i},SV\right)lgQ\left(F_{i},SV\right)}$, [1] so the computational cost is linear. The time complexity is *P*(*n*). Secondly, the information loss metric needs to be calculated: Qre(*ST*)=1 − ∑_*i*=1_^*N*^∑_*j*=1_^*N*_*A*_^*h*/|DGH_*Bi*_|/*N∗N*_*A*_, and there are two cumulative multiplication operations in the calculation process, so the calculation overhead at this stage is *P*(^*n*2^). Finally, the attributes need to be processed at the domain generalization level. The computational cost of each generalization is linear, so the computational complexity is *P*(*n*).

### 5.3. Execution Time Analysis

It can be seen that Figure 1 with Table 7 shows that as the number of RIs increases, the execution time of the three models will increase. This is because as the RI value increases, the equivalence class also rises.

More quasi-identifier attributes must be recorded, which requires more generalization times. This process also requires the algorithm to execute more cycles to increase the execution time.

At the same time, it can be seen that as the QI value increases, the execution time of the proposed scheme is shorter than that of the information entropy *l*-diversity model. This is because it takes longer for the information entropy *l*-diversity model to judge the strong and weakly sensitive attributes in the equivalence class.

Figure 2 with Table 8 describes the change of data accuracy with the value of *k* or *l* in the three anonymous models when QI records increase from 0 to 1,000. The abscissa is the number of documents, and the ordinate is the time to execute different algorithms. It can be seen that the solution in this paper improves the data accuracy while reducing the execution time of the algorithm.

### 5.4. Precision Analysis

Figure 3 with Table 9 describes the change of data accuracy with the value of *k* or *l* in the three anonymous models when QI records increase from 1,000 to 3,500. The abscissa is the number of documents, and the ordinate is the data accuracy of the unknown dataset. It can be found that as the number of records increases, the accuracy of this solution is higher than other solutions.

### 5.5. Information Loss Analysis

Figure 4 with Table 10 describes the change of data accuracy with the value of *k* or *l* in the three anonymous models when the number of QIs is 0–8. The abscissa is the value of *k* and *l*, and the ordinate is the data accuracy of the anonymous dataset.

Figure 3 describes as the values of *k* and *l* increase, the accuracy of the data shows a downward trend. As the importance of *k* and *l* increases, the number of tuples that need to be generalized in the equivalence class increases. The higher the generalization level, the greater is the information loss, and the data accuracy will decrease. Under the same circumstances, the information loss of personalized information entropy *l*-diversity is higher than that of information entropy *l*-diversity. This is because customized information entropy *l*-diversity has more substantial constraints on anonymity than information entropy *l*-diversity. Higher-level generalization needs to be aligned with the identifier, so the information loss is relatively significant.

## 6. Conclusion

Aiming at the problem that the information entropy *l*-diversity model does not distinguish between strong and weak sensitive attributes, this paper proposes a personalized information entropy *l*-diversity model and conducts experiments. The privacy of the proposed model is better than other models. Because it secures personal data while preserving data availability, k-anonymity, based on the incognito principle, has become an essential technical technique for privacy protection in data release. The basic concept is to use generalizations and concealing methods to publish data with low accuracy. Each record in the datasheet has at least the same quasi-identifier attribute value as the other *k* − 1 data in the database, decreasing security leaks caused by connection threats. The drawback of the proposed algorithm is that erroneous query results throughout the calculating process, especially when users are scarce. It will also create a broader anonymous area, which will increase the communication overhead. The experimental results show that the performance of this solution in terms of execution time and data accuracy is better than the information entropy l-diversity model and k-anonymity model, and it has better privacy. It can be used in mobile medical systems to protect medical users. Private data will not be leaked. The scope of this research is that the data analysis and trial findings reveal that this strategy is more effective than previous alternatives in terms of reducing execution time while boosting data accuracy and service quality.

## Figures and Tables

**Figure 1:** Comparison of execution time with the number of quasi identifiers.

**Figure 2:** Comparison of execution time with the number of records.

**Figure 3:** Comparison of data accuracy with the number of records.

**Figure 4:** Comparison of data accuracy with *l*, *k* value.

**Table 1:** The sheet of medical data.

Age	Sex	Zip	Disease
22	F	103658	Short breath
24	M	158083	Influenza
25	M	158086	Fever
27	F	350186	Insomnia
29	M	213045	Influenza
33	F	120654	Hepatitis
35	M	430056	Obesity
36	M	131548	Emphysema

**Table 2:** The list of voter poll.

Name	Age	Sex	Zip	Party
Tim	25	M	132635	Member
Linda	28	F	151346	N/a
Kevin	35	M	430056	Member
Mary	37	F	350186	Member

**Table 3:** The meeting 2- anonymous data sheet.

Age	Sex	Zip	Disease
(20, 30]	M	1211^*∗∗*^	Pneumonia
(20, 30]	M	1211^*∗∗*^	Influenza
[30, 40]	F	1315^*∗∗*^	Diabetes
[30, 40]	F	1315^*∗∗*^	Diabetes
(40, 50]	^*∗*^	1526^*∗∗*^	Heart disease
(40, 50]	^*∗*^	1526^*∗∗*^	Hypertension

^*∗*^ signifies the approximate value.

**Table 4:** The meeting 5- anonymous equivalence class.

Age	Sex	Zip	Disease
(20, 30]	M	1236^*∗∗*^	Influenza
(20, 30]	M	1236^*∗∗*^	Influenza
(20, 30]	M	1236^*∗∗*^	Influenza
(20, 30]	M	1236^*∗∗*^	Diabetes
(20, 30]	M	1236^*∗∗*^	Influenza

^*∗∗*^ signifies the approximate value.

**Table 5:** The structure of Adult dataset.

Attributes	Difference value	Weights
Age	74	4
Gender	2	2
Race	5	2
Educate	16	4
Employer	7	3
Country of citizenship	41	3
Profession	14	2
Disease	10	—

**Table 6:** The weight of disease.

Numbering	Disease	Weights
**1**	Influenza	0.11
**2**	Obesity	0.12
**3**	Fever	0.13
**4**	Angrily kick	0.31
**5**	Insomnia	0.41
**6**	Chest pain	0.42
**7**	Hepatitis	0.51
**8**	Myocarditis	0.91
**9**	Tuberculosis	0.92
**10**	Depression	0.93

**Table 7:** Comparison of execution time with the number of quasi identifiers.

S. No.	*l*-diversity	*l*-diversity	k-diversity
30	50	60	70
40	55	65	75
50	80	90	100
60	130	140	150
70	230	240	250

**Table 8:** Comparison of execution time with the number of records.

S. No.	*l*-diversity	*l*-diversity	k-diversity
200	50	60	70
400	55	65	75
600	100	150	200
800	250	300	350
1000	400	380	500

**Table 9:** Comparison of data accuracy with the number of records.

S. No.	*l*-diversity	*l*-diversity	k-diversity
1000	0.72	0.73	0.74
1500	0.725	0.735	0.745
2000	0.73	0.735	0.74
2500	0.745	0.75	0.755
3000	0.755	0.76	0.765
3500	0.76	0.768	0.77

**Table 10:** Comparison of data accuracy with *l*, *k* value.

S. No.	*l*-diversity	*l*-diversity	k-diversity
2	0.8	0.78	0.75
3	0.7	0.73	0.7
4	0.65	0.6	0.64
5	0.6	0.55	0.58
6	0.5	0.4	0.45
7	0.25	0.29	0.3

## Data Availability

The data shall be made available on request.

## References

[1] Tripathy B. K., Maity A., Ranajit B., Chowdhuri D. A fast p-sensitive l-diversity Anonymisation algorithm.

[2] Zhu H., Tian S., Lu K. (2015). Privacy-preserving data publication with features of independent -diversity. *The Computer Journal*.

[3] Han Jianmin J., Cen Tingting T., Yu Juan J. An l-MDAV microaggregation algorithm for sensitive attribute l-diversity.

[4] Enam M. A., Sakib S., Rahman M. S. An algorithm for l-diversity clustering of a point-set.

[5] Testard M., Nivelet J. C., Matos T., Levannier G. (1997). Tight approximation of bit error probability for L-diversity non-coherent M-ary FSK frequency hopping system with binary convolutional code and soft Viterbi decoder: diversity, bit interleaver size and Reed-Solomon outer code effects analysis on receiver performance for M=8. *MILCOM 97 MILCOM 97 Proceedings*.

[6] Jianmin Han J., Huiqun Yu H., Yu J. An improved l-diversity model for numerical sensitive attributes.

[7] Xiao H.-L., Ouyang S., Nie Z.-P. Design and performance analysis of compact planar inverted-L diversity antenna for handheld terminals.

[8] Tripathy B. K., Mitra A. An algorithm to achieve k-anonymity and l-diversity anonymisation in social networks.

[9] Miyakawa S., Saji N., Mori T. Location l-diversity against multifarious inference attacks.

[10] Mehbodniya A., Alam I., Pande S. (2021). Financial fraud detection in healthcare using machine learning and deep learning techniques. *Security and Communication Networks*.

[11] Tiwari A., Dhiman V., Iesa M. A. M., Alsarhan H., Mehbodniya A., Shabaz M. (2021). Patient behavioral analysis with smart healthcare and IoT. *Behavioural Neurology*.

[12] Temuujin O., Ahn J., Im D.-H. (2019). Efficient L-diversity algorithm for preserving privacy of dynamically published datasets. *IEEE Access*.

[13] Gong L., Guo F., Miao Q., Li H., Jie W., Zhang W. Location privacy protection in mobile social networks based on l-diversity.

[14] Gaoming Yang G., Jingzhao Li J., Li Yu S., Yu Li An enhanced l-diversity privacy preservation.

[15] Soni M., Singh D. K. (2021). LAKA: lightweight Authentication and key agreement protocol for internet of things based wireless body area network. *Wireless Personal Communication*.

[16] Ghozali M., Satibi S., Ikawati Z., Lazuardi L. (2021). Asthma self-management app for Indonesian asthmatics: a patient-centered design. *Computer Methods and Programs in Biomedicine*.

